The article "Effects of Silicone Mattress Combined with Hydrocolloid Dressing on Pressure Ulcers and Phlebitis in ICU Patients with Liver Failure" was retracted in 2023. Reasons: unreliable results or conclusions; concerns about the data; concerns about the peer review; concerns about the citations.

# Effects of Silicone Mattress Combined with Hydrocolloid Dressing on Pressure Ulcers and Phlebitis in ICU Patients with Liver Failure

**DOI:** 10.1155/2022/7828650

**Published:** 2022-04-15

**Authors:** Suhong Chen, Yonggang Wang, Shun Huang, Dan Wu, Yinyin Li, Zhiqiang Zhong, Yajin Xue, Huanxin Li, Jinsong Mu

**Affiliations:** ^1^Department of Critical Care Medicine, The Fifth Medical Center of Chinese PLA General Hospital, 100039 Beijing, China; ^2^Nursing Department, The Fifth Medical Center of Chinese PLA General Hospital, 100039 Beijing, China; ^3^Infectious Disease Department, The Fifth Medical Center of Chinese PLA General Hospital, 100039 Beijing, China; ^4^Department of Liver Disease, The Fifth Medical Center of Chinese PLA General Hospital, 100039 Beijing, China

## Abstract

**Objective:**

This study was aimed at clarifying the application effect of silicone mattress combined with hydrocolloid dressing in ICU patients with liver failure.

**Methods:**

A total of 86 patients with liver failure admitted to the intensive care unit (ICU) of the Fifth Medical Center of Chinese PLA General Hospital from September 2018 to September 2020 were selected as the research subjects. Patients treated with conventional sponge mattress and routine nursing care were included in group A (*n* = 43), and those treated with silicone mattress combined with hydrocolloid dressing were included in group B (*n* = 43). The incidence of pressure ulcers and phlebitis, the scores of Visual Analogue Scale (VAS) and Pittsburgh Sleep Quality Index (PSQI), and the nursing satisfaction were observed and compared between the two groups.

**Results:**

The incidence of pressure ulcers in group B (6.98%) was lower than that in group A (25.58%). The incidence of phlebitis in group B was lower than that in group A (20.93% vs. 53.49%). The VAS score of group B was 2.16 ± 0.38, which was lower than that of group A (4.86 ± 1.09). The PSQI score of group B was lower than that of group A (9.74 ± 2.76 vs. 14.84 ± 3.95). A higher nursing satisfaction was determined in group B compared with group A (93.02% vs. 76.74%).

**Conclusions:**

Silicone mattress combined with hydrocolloid dressing can reduce the incidence of pressure ulcers and phlebitis in ICU patients with liver failure, reduce complications, and improve nursing satisfaction, which is worthy of clinical promotion.

## 1. Introduction

Liver failure (LF) is manifested as a group of serious clinical symptoms such as jaundice, coagulation dysfunction, hepatorenal syndrome, hepatic encephalopathy, and ascites [1]. In China, LF is mainly caused by hepatitis virus (especially hepatitis C virus), while drugs and hepatotoxic substances (alcohol, chemicals, etc.) are secondary causes. LF in children can also be caused by genetic metabolic diseases. Both acute and subacute LF are acute episodes with no underlying medical history. The clinical manifestations of LF are acute within 2 weeks of onset and subacute between 2 and 26 weeks. At present, there is no consensus on the definition of acute-on-chronic liver failure (ACLF), but it is generally considered to be a short-term sudden onset of liver decompensation and LF on the basis chronic liver failure (CLF). According to the literature, 75% to 90% of domestic LF is ACLF [2]. CLF is based on liver cirrhosis, which is mainly manifested as hepatic encephalopathy caused by slow liver dysfunction and can only be treated by liver transplantation. It has been reported [3] that the fatality rate of LF is 73.9%. The worse the coagulation function, the higher the fatality rate. Therefore, studying the management strategy of LF in ICU patients has important practical significance for reducing patient mortality, which is also the purpose of this study.

The article "Effects of Silicone Mattress Combined with Hydrocolloid Dressing on Pressure Ulcers and Phlebitis in ICU Patients with Liver Failure" was retracted in 2023. Reasons: unreliable results or conclusions; concerns about the data; concerns about the peer review; concerns about the citations.

Studies have calculated that since the establishment of intensive care unit (ICU) service for liver diseases, the survival rate of patients with LF has increased from 21% to about 58%, indicating that timely and effective ICU treatment is beneficial to improve the survival of critically ill patients [4]. Acute and subacute LF patients have fast onset and rapid development. Therefore, such patients should be immediately transferred to ICU for monitoring and treatment when they develop symptoms of hepatic encephalopathy. In addition, critically ill patients are prone to skin breakage and pressure ulcers due to edema, weight loss, and inability to turn over after admission to ICU. Pressure ulcer, which is one of the most common complications in ICU patients with LF, refers to local tissue necrosis caused by tissue hypoxia due to long-term local tissue compression, malnutrition, and obstructed blood circulation [5]. As for the treatment, three-way valve peripherally inserted central catheter (PICC) catheterization is a deep vein operation technique for patients with LF. However, as a foreign body in direct contact with the outside world, improper care, improper operation, or long-term high concentration of strong irritating drugs can easily cause adverse reactions in patients, among which phlebitis is the most common [6]. There are four main types of phlebitis, namely, mechanical phlebitis, chemical phlebitis, infectious phlebitis, and thrombophlebitis [7]. Studies have shown that 3% to 30% of patients receiving intravenous indwelling needle infusion have phlebitis of varying degrees [8].

Routine care is usually to give ECG monitoring and oxygen inhalation to patients with LF after entering the ICU and to observe the vital signs of patients. The care usually involves gentle operation to avoid skin damage, the use of an air bed to help the patient turn over, changing sheets in a timely manner, and keeping the patient's skin clean [9]. In addition, 50% magnesium sulfate wet compress is often used to treat phlebitis; however, the gauze is easy to harden and fall off when applied externally, and high-concentration magnesium sulfate is easy to form crystals and pollute sheets [10]. It can be seen that these nursing methods can reduce pressure ulcers and phlebitis to a certain extent, but the effect is not ideal. Therefore, effective nursing measures are needed to reduce the occurrence of pressure ulcers and phlebitis in patients.

The article "Effects of Silicone Mattress Combined with Hydrocolloid Dressing on Pressure Ulcers and Phlebitis in ICU Patients with Liver Failure" was retracted in 2023. Reasons: unreliable results or conclusions; concerns about the data; concerns about the peer review; concerns about the citations.

The silicone mattress is a mattress made of a new type of semisolid material, whose outer layer is wrapped with a silicone layer and the inner layer is silicone gel [11]. This kind of mattress has no fluidity, good flexibility, and pressure resistance, which can be naturally shaped according to the contour of the human body; in addition, its surface is smooth, waterproof, and antipollution, which allows for repeated uses after disinfection without harming the human skin; moreover, it has excellent airtightness, X-ray transmission, and static electricity. In pressure ulcer-prone areas, such as bone protuberances, the use of silicone mattress can evenly distribute the patient's mass and increase the area of force, which can effectively reduce the pressure, shear, and friction per unit area of the body surface to avoid skin damage and the formation of pressure ulcers.

The hydrocolloid dressing is composed of calcium alginate, sodium carboxymethyl cellulose, pectin, and hydropeptide microparticle gelatin. It is divided into an inner layer and an outer layer. The outer layer is a polyurethane semipermeable membrane, and the inner layer consists of polymeric hydrogels as well as synthetic rubber and adhesives [12]. This design can prevent microbial invasion while reducing water loss and maintaining a moist environment. In addition, its double viscosity can promote cell proliferation and epithelial collagen synthesis, which is conducive to facilitating the growth of microvessels and repairing vascular endothelial cells. The hypoxic tension formed by the skin also helps to accelerate the resolution of inflammation [13]. However, there are currently no reports on the application of silicone mattress combined with hydrocolloid dressing in ICU patients with LF. Therefore, this study reported for the first time the application effect of the combination treatment of silicone mattress and hydrocolloid dressing in ICU hospitalized LF patients.

The article "Effects of Silicone Mattress Combined with Hydrocolloid Dressing on Pressure Ulcers and Phlebitis in ICU Patients with Liver Failure" was retracted in 2023. Reasons: unreliable results or conclusions; concerns about the data; concerns about the peer review; concerns about the citations.

## 2. Materials and Methods

### 2.1. General Information

In this study, 86 patients with LF admitted to the ICU of the Fifth Medical Center of Chinese PLA General Hospital from September 2018 to September 2020 were selected and divided into group A (*n* = 43) and group B (*n* = 43). Inclusion criteria are as follows: (1) in accordance with the clinical diagnostic criteria for LF; (2) no history of antiviral drug treatment; (3) expected hospital stay ≥ 1 week; (4) and voluntarily participation in the study with informed consent provided. Exclusion criteria are as follows: (1) autoimmune hepatitis or genetic metabolic diseases; (2) death within 1 week of hospitalization; and (3) inability to cooperate due to unconsciousness. In group A, there were 23 males and 20 females, with an average age of 55.49 ± 4.26 years and a mean admission time of 10.76 ± 1.81 days. In group B, there were 30 males and 13 females, with an average age of 56.17 ± 3.02 years and a mean hospitalization time of 10.92 ± 1.78 days. The comparison of general information revealed no significant difference between the two groups (*P* > 0.05), indicating comparability. The study was approved by the Ethics Committee of the Fifth Medical Center of Chinese PLA General Hospital.

### 2.2. Methods

#### 2.2.1. Group A

Patients in group A were treated with conventional foam mattress and routine nursing care, specifically as follows. Before the operation, the risk of intraoperative pressure ulcers was determined, and appropriate operating beds and bed sheets were selected for patients. In addition, patients were instructed to keep their clothing dry. During the operation, the patient's skin was closely monitored and managed, and the body temperature and skin surface temperature were controlled. The pressure ulcer risk assessment was performed again after the operation. Finally, sponge pads were given to patients at the site prone to pressure ulcers for prevention. Thick, straight, flexible, and easy-to-puncture forearm blood vessels were selected for observation, and attention was paid in avoiding the venous valves and veins near joints, as well as inflammatory and indurated veins. A three-way valve PICC catheter was used and fixed conventionally. See Figure 1 for the silicone mattress.

#### 2.2.2. Group B

Patients in group B were treated with silicone mattress combined with hydrocolloid dressing. On the basis of routine care in group A, silicone mattress (ACTION Company, USA) was used in group B. After successful puncture, patients were covered with hydrocolloid dressings (ConvaTec Inc, 211 American Avenue, Greensboro, North Carolina 27409, USA) over the puncture point of the indwelling needle in addition to routine fixation, and the indwelling needle was removed at the end of the drug infusion, leaving the hydrocolloid dressings for 1 d. See Figure 2 for the hydrocolloid dressing.

The article "Effects of Silicone Mattress Combined with Hydrocolloid Dressing on Pressure Ulcers and Phlebitis in ICU Patients with Liver Failure" was retracted in 2023. Reasons: unreliable results or conclusions; concerns about the data; concerns about the peer review; concerns about the citations.

### 2.3. Observation Indicators

#### 2.3.1. Staging of Pressure Ulcers

Staging criteria for pressure ulcers are as follows [14]: Stage IV: exposed tendons, muscles, and bones, with tissue crusting, shedding, undermining, or tunneling. Stage III: full-thickness skin loss, visible subcutaneous adipose tissue, with tissue shedding and necrosis, but no exposed tendons, muscles, and bones, with or without the presence of undermining and tunneling. Stage II: skin, dermis, and epidermis damage, pink wound bed, and symptoms of congestive blisters or rupture of ulcers. Stage I: intact skin surface, but the part of the skin appears red; the color does not fade when pressed with the fingers and differs significantly from the surrounding area. The incidence of pressure ulcers = (stage I + stage II + stage III + stage IV) cases/total number of cases × 100%.

#### 2.3.2. Grading of Phlebitis

Grading criteria for phlebitis are as follows [15]: Grade 0: asymptomatic. Grade 1: slight redness at the puncture site with or without pain. Grade 2: pain, redness, and/or edema at the puncture site. Grade 3: pain, redness, and/or edema at the puncture site, with cord-like structure formation and palpable cord veins. Grade 4: pain at the puncture site, accompanied by congestion and/or edema, formation of cord-like structure, palpable cord veins (length > 2.5 cm), and pus exudation. The incidence of phlebitis was calculated as the percentage of total cases except grade 0 in the total cases.

#### 2.3.3. Pain Score and Sleep Quality Score

All patients were scored for pain severity and sleep quality 1 week after the operation. The degree of pain was scored using the Visual Analogue Scale (VAS) [16]. A 10 cm ruler was used, with each 1 cm representing 1 point and a total score of 10 points. 0 indicates painless, and a score of 10 points indicates unbearable pain. All patients were instructed by their doctors to determine their own pain levels and their scores were recorded to two decimal places. The sleep quality of patients was evaluated using the Pittsburgh Sleep Quality Index (PSQI) [17]. The scale has 7 dimensions (18 items), and each dimension is divided into 0 to 3 levels, with a total score of 21 points. The higher the score, the worse the quality of sleep. In addition, the scale has 5 other rated items and 19 self-rated items, which can assist in judging the patient's sleep quality, but does not score.

The article "Effects of Silicone Mattress Combined with Hydrocolloid Dressing on Pressure Ulcers and Phlebitis in ICU Patients with Liver Failure" was retracted in 2023. Reasons: unreliable results or conclusions; concerns about the data; concerns about the peer review; concerns about the citations.

#### 2.3.4. Nursing Satisfaction

Nursing satisfaction was assessed using the self-made questionnaire of our hospital, with 25 items in total and 4 points for each item. On a 100-point scale, a score of ≥80 points indicates very satisfied, 60-80 indicates satisfied, and <60 points indicates unsatisfactory. Nursing satisfaction = (very satisfied + satisfied) cases/total number of cases × 100%.

### 2.4. Statistical Methods

The SPSS 22.0 (SPSS Inc., Chicago, IL, USA) was used for statistical analysis. Quantitative data is expressed as (^−^x ± s), and qualitative data is expressed as *n* (%). The statistical methods for ordered qualitative data (e.g., pressure ulcer staging and phlebitis grading), disordered qualitative data (e.g., nursing satisfaction), and quantitative data (e.g., VAS and PSQI scores) were rank sum test, *χ*^2^ test, and *t* test, respectively. *P* < 0.05 indicates that the difference was statistically significant.

## 3. Results and Discussion

### 3.1. Comparison of the Occurrence of Pressure Ulcers between the Two Groups

In group A, there were 6 cases of pressure ulcers in stage I, 3 cases in stage II, and 2 cases in stage III; in group B, 2 cases had stage I pressure ulcers and 1 case had stage II pressure ulcer. The incidence of pressure ulcers in group B was lower than that in group A (6.98% vs. 25.58%; *χ*^2^ = 4.181, *P* = 0.041; Figure 3).

### 3.2. Comparison of the Occurrence of Phlebitis between the Two Groups

Group A has 20 cases of grade 0 phlebitis, 12 cases of grade 1, 8 cases of grade 2, 2 cases of grade 3, and 1 case of grade 4; group B has 34 cases of grade 0 phlebitis, 5 cases of grade 1, 3 cases of grade 2, 3 cases of grade 3 1 case, and 0 cases of grade 4. The incidence of phlebitis in group B was 20.93%, which was lower than that in group A 53.49% (*Z* = −5.055, *P* < 0.001; Figure 4).

### 3.3. Comparison of VAS Score and PSQI Score between the Two Groups

The VAS score of group B (2.16 ± 0.38) was lower than that of group A (4.86 ± 1.09) (*t* = 15.341, *P* < 0.001, Figure 5(a)); a lower PSQI score was also determined in group B compared with group A (9.74 ± 2.76 vs. 14.84 ± 3.95; *t* = 6.940, *P* < 0.001, Figure 5(b)).

### 3.4. Comparison of Nursing Satisfaction between the Two Groups

In group A, 18 cases were very satisfied, 15 cases were satisfied, and 10 cases were dissatisfied. In group B, 33 cases were very satisfied, 7 cases were satisfied, and 3 cases were dissatisfied. The nursing satisfaction rate of group B was higher than that of group A (93.02% vs. 76.74%; *Z* = −4.436, *P* < 0.001; Figure 6).

## 4. Discussion

Pressure ulcers are a very common complication in clinical care, mainly due to the injury caused by other primary diseases in the treatment process and the poor management of the diseases. This is particularly true for patients with severe LF, as they may lie down for a long time due to malnutrition, weight loss, and other reasons, resulting in the difficulty in turning over and higher susceptibility to pressure ulcers. When pressure ulcers occur, the skin usually ruptures, which increases the pain of severe patients, reduces their sleep quality and life quality, prolongs the recovery time, and increases the medical cost. In addition, the skin, as the first line of defense for immunity, is more likely to induce wound infections when the immune function of severely ill patients is weak.

The article "Effects of Silicone Mattress Combined with Hydrocolloid Dressing on Pressure Ulcers and Phlebitis in ICU Patients with Liver Failure" was retracted in 2023. Reasons: unreliable results or conclusions; concerns about the data; concerns about the peer review; concerns about the citations.

The risk factors of pressure ulcers include local as well as systemic factors [18]. Local factors are mainly due to local pressure, tissue shear stress, skin friction, and skin moisture [19]. Pressure is the most direct cause of pressure ulcers. Long-term bed rest refers to the condition in which most of the skin of the body, especially the sacrococcygeal and buttocks in the supine position, the sacrococcygeal area in the semisitting position and the shoulders and buttocks in the lateral position are subjected to pressure. This state will cause skin pressure and obstruction and disorder of the microvascular circulation, leading to local tissue ischemia and hypoxia as well as nutrient supply deficiency and necrosis, ultimately inducing pressure ulcers.

It is believed that tissue damage is closely related to the level of pressure and the duration of compression [20]. If it exceeds 9.3 k Pa for 2 hours, it can cause irreversible damage to tissue cells. In the percolating tissue, the soft tissue is affected by the shear force to produce relative transverse displacement, which will twist the deep blood vessels of the superficial fascia. If the twist is too long for too long a time, it can make the blood supply insufficient in a larger area, leading to microthrombosis and reduced tissue oxygen tension. Shear forces are more harmful and can cause irreversible damage to deep tissues within 30 minutes, but the signs of skin surface damage may not be obvious or even visible. The impact of shear forces on blood vessels and blood circulation is more harmful than pressure. When both exist, the incidence of pressure ulcers is higher.

When friction and skin epithelial tissues rub against each other, the outer layer of the skin will protect the stratum corneum, causing the increase of local skin temperature, tissue metabolism, and oxygen consumption. Pressure ulcers are more likely to occur in compressed, ischemic, and hypoxic tissues. Friction is present in many settings, especially when there are wrinkles and residues on the surface of the sheet. In addition, there will be greater friction when the patient moves. In addition to the above factors, a moist skin environment can also promote the formation of pressure ulcers. Systemic factors include malnutrition, age, and psychological factors, among which malnutrition is considered the internal cause of pressure ulcers and the second risk factor for pressure ulcers after stress. Malnutrition causes a decline in immune function and stress metabolism regulation, muscle atrophy, and loss of subcutaneous fat. The compressed local skin tissue lacks the protection of muscle and fat, with weakened ability to withstand pressure, which is more likely to cause local blood circulation disorders and pressure ulcers.

The article "Effects of Silicone Mattress Combined with Hydrocolloid Dressing on Pressure Ulcers and Phlebitis in ICU Patients with Liver Failure" was retracted in 2023. Reasons: unreliable results or conclusions; concerns about the data; concerns about the peer review; concerns about the citations.

Elderly patients with LF are more likely to develop pressure ulcers because of loose skin, lack of support and elasticity, slow metabolism, and difficulty in recovery after damage. The material characteristic of the silicone mattress is that the patient's mass is evenly distributed on the mattress. According to the principle of the force area, the force per unit area is greatly reduced after the uniform distribution. The first thing to reduce the pressure is to reduce the pressure directly so that the local circulation is no longer blocked and the skin can flow smoothly. The use of the mattress can effectively adjust the shearing force and avoid deep tissue damage. In addition, the smooth surface of the material greatly avoids the threat of friction. As shown in Figure 3, the incidence of pressure ulcers in group B (6.98%) was lower than that in group A (25.58%). This shows that the silicone mattress has a significant effect on the prevention of pressure ulcers, which can reduce the incidence of pressure ulcers, facilitate patient recovery and pain relief, and improve their sleep quality.

The three-way valve PICC catheterization is a method of central venous insertion of a three-way valve catheter through peripheral vascular puncture. Due to the high success rate of catheterization and favorable safety, it has been widely used in the care of ICU patients with LF [21]. But it can easily cause phlebitis. This may be due to mechanical damage during venous catheterization, allergic reactions caused by catheter materials, environmental pollution during puncture, and drug injection stimulation [22]. In the process of venous catheterization, the stimulation of the blood vessel wall will cause vasoconstriction. At the same time, the resistance of the venous valve and the bypassing part of the blood vessel may cause damage to the blood vessel wall, and the inflammatory substances released after the injury may be closed to form local inflammatory edema. Although the catheter is made of nonallergenic high-grade silicone materials, the human body's immune rejection of foreign bodies can still cause inflammation. And if the puncture site is not properly disinfected and the environmental particles are not cleaned up, it is easy to cause phlebitis. Critically ill patients may be given drugs that are more irritating, which may stimulate blood vessels and surrounding tissues. Hydrocolloid dressings, which are composed of elastic polymer hydrogels, synthetic rubbers, and viscous materials, can absorb exudate, with good airtightness to prevent microbial invasion. In addition, they maintain a moist environment and are excellent for cleansing. Moreover, they can promote the synthesis of epithelial collagen, repair the damaged blood vessel wall, generate capillary blood vessels, and increase capillary perfusion. Therefore, they play a significant role in the prevention and treatment of phlebitis. In this study, the incidence of phlebitis in group B was 20.93%, which was lower than that in group A (53.49%), indicating the good performance of hydrocolloid dressings in the prevention of phlebitis.

The article "Effects of Silicone Mattress Combined with Hydrocolloid Dressing on Pressure Ulcers and Phlebitis in ICU Patients with Liver Failure" was retracted in 2023. Reasons: unreliable results or conclusions; concerns about the data; concerns about the peer review; concerns about the citations.

The results of this study indicated that compared with group A, the incidence of pressure ulcers and phlebitis in group B was significantly lower, the relief of pain and sleep disorders was significantly better, and the nursing satisfaction was significantly higher. This indicates that silicone mattress combined with hydrocolloid dressing has a significant impact on ICU patients with LF, which can reduce complications and promote rehabilitation. In addition, the novelty of this study lies in the analysis and verification of the efficacy and safety of silicone mattress combined with hydrocolloid dressing in ICU patients with LF from multiple aspects such as the occurrence of pressure ulcers and phlebitis, pain, sleep quality, and nursing satisfaction, providing a new choice for the clinical management of LF patients hospitalized in ICU.

## 5. Conclusion

This study is the first to report the application value of silicone mattress combined with hydrocolloid dressing in ICU patients with LF. It was found that silicone mattress can significantly reduce the incidence of pressure ulcers in ICU patients with LF, and hydrocolloid dressing is highly effective in preventing phlebitis, indicating that silicone mattress combined with hydrocolloid dressing can be used in ICU patients with LF. Therefore, this study argues that the combined treatment has remarkable clinical application value and is worthy of clinical promotion in the treatment of ICU patients with LF, as it can reduce complications, promote rehabilitation, and improve nursing comfort and satisfaction.

The article "Effects of Silicone Mattress Combined with Hydrocolloid Dressing on Pressure Ulcers and Phlebitis in ICU Patients with Liver Failure" was retracted in 2023. Reasons: unreliable results or conclusions; concerns about the data; concerns about the peer review; concerns about the citations.

## Figures and Tables

**Figure 1:** Silicone mattress.

**Figure 2:** Hydrocolloid dressing.

**Figure 3:** Comparison of the occurrence of pressure ulcers between the two groups.

**Figure 4:** Comparison of the occurrence of phlebitis between the two groups.

**Figure 5:** Comparison of VAS score and PSQI score between the two groups. (a) Comparison of the VAS scores between the two groups. (b) Comparison of PSQI scores between the two groups. ^∗∗∗^*P* < 0.001.

**Figure 6:** Comparison of nursing satisfaction between the two groups.

## Data Availability

The labeled datasets used to support the findings of this study are available from the corresponding author upon request.
